# Evaluation Value and Clinical Significance of Cardiac Troponin Level and Pediatric Sequential Organ Failure Score in the Definition of Sepsis 3.0 in Critically Ill Children

This article has been retracted.

**DOI:** 10.1155/2022/9492178

**Published:** 2022-08-09

**Authors:** YunDuo Wu, Wenli Shen, Qizheng Wang, Changqiang Cui, Li Zha, Yan Jiao Lu, Rui Liu, Xiaofei Lin, Hongli Zhu

**Affiliations:** ^1^Department of Pediatrics, Huai'an Maternal and Child Health Care Hospital, Huaian, Jiangsu, China 223002; ^2^Department of Pediatrics, Xuyi People's Hospital, Huaian, Jiangsu, China 223400

## Abstract

**Objective:**

A case-control study was conducted to explore the value and clinical significance of troponin level and pediatric sequential organ failure score in the evaluation of sepsis 3.0 definition in critically ill children.

**Methods:**

180 children with sepsis who were admitted to the ICU from March 2019 to June 2021 were enrolled in our hospital as the research objects. In addition, 100 children with general infection did not meet the diagnostic criteria of systemic inflammatory response syndrome (SIRS) as controls. The creatine kinase MB (CK-MB) and cardiac troponin I (cTnI) data at the 1st and 24-72 h after admission to pediatric intensive care unit (PICU) were enrolled as the observation indexes of myocardial enzymology. In the meantime, the relevant literature was reviewed to obtain the indicators related to sepsis death. The data of the first examination in the medical history data were enrolled for analysis. According to the definition of sepsis 3.0 in critically ill children, they were assigned into sepsis and nonsepsis group. According to the survival outcome of discharge and 30 days after discharge, the patients were assigned into the death subgroup and survival subgroup and were assigned into the sequential organ failure assessment (SOFA) score ≥ 2 subgroup and< 2 subgroup according to SOFA score. COX proportional hazard regression was used to analyze the relationship between CK-MB, cTnI, and SOFA scores and prognosis. ROC curve was adopted to analyze the value of CK-MB, cTnI, and SOFA scores in the evaluation of critical sepsis in children.

**Results:**

Univariate analysis indicated that the prognosis of children with sepsis was correlated with abnormal levels of CK-MB and cTnI, SOFA score, oxygenation index < 200, mean arterial pressure, and Glasgow coma scale (GCS), and the difference was statistically significant (*P* < 0.05). The results of COX regression analysis indicated that the variables that were remarkably associated with death from sepsis in children were CK-MB, elevated cTnI levels, and SOFA score ≥ 2, and serum cTnI and/or CK-MB levels and SOFA score were remarkably higher correlation (*r* = 0.453, *P* < 0.05). In terms of the myocardial enzyme levels in the sepsis group and the nonsepsis group, the levels of CK-MB and (or) cTnI augmented in 121/180 cases (67.22%) in the sepsis group and in 19/100 cases (19.00%) in the nonsepsis group. The levels of CK-MB and (or) cTnI were augmented, and the difference was statistically significant (*P* < 0.05). The levels of CK-MB and cTnI in the sepsis group at admission to ICU and 24 to 72 hours after admission were remarkably higher compared to the nonsepsis group. The levels of CK-MB and cTnI at 24-72 h were higher compared to ICU. The myocardial enzyme levels of different SOFA scores and survival outcome subgroups in the sepsis group were compared. The subgroup with SFOA score ≥ 2 points had remarkably higher levels of CK-MB and (or) cTnI than the subgroup with <2 points. The survival subgroup of CK-MB and cTnI level was remarkably higher compared to the death subgroup, the CK-MB and cTnI levels in each subgroup at 224-72 hours were remarkably higher compared to the ICU, and the difference was statistically significant (*P* < 0.05). Kaplan-Meier method and log-rank test indicated that the survival rates of groups 1 to 4 at 30 days were 33.23%, 78.71%, 40.03%, and 100.00%, respectively. The average survival time and their 95% CI were 12.82 d (10.52~ 16.26 d), 22.34 d (18.76~ 25.81 d), 14.65 d (11.62~ 16.38 d), and 30 d (30.00~ 30.00 d), respectively. Pairwise comparison indicated that the survival time of children in group 1 was the shortest, and that in group 4 was the longest. The results of ROC curve research showed that the CK-MB, cTnI, and SOFA scores and AUC for the combination test were 0.778 (95% CI 0.642–0.914), 0.736 (95% CI 0.602–0.890), 0.848 (95% CI 0.733–0.963), and 0.934 (95% CI 0.854–0.999), respectively. The AUC of combined diagnosis was remarkably higher compared to single factor prediction, and the difference was statistically significant (*P* < 0.05). Predictive value showed the joint test > SOFA score > CK − MB > cTnI.

**Conclusion:**

Troponin level and pediatric SOFA score can be adopted as effective indicators to assess the severity and prognosis of patients with sepsis and can guide the formulation of a reasonable treatment plan.

## 1. Introduction

The definitions and standards of childhood sepsis and septic shock were first proposed at the 2004 International Childhood Sepsis Consensus Conference in San Diego, USA, to raise awareness of sepsis [1]. Since then, the guidelines in 2008 and 2012 have made recommendations for new diagnosis and treatment of sepsis. Sepsis is a systemic inflammatory response syndrome caused by an infection (suspected/confirmed), i.e., fever (anal temperature > 38.5°C) or hypothermia (anal temperature < 35°C), accompanied by at least one of the following abnormalities: flooding of the pulse, altered consciousness, hypoxemia, and elevated serum lactate [2]. Septic shock refers to cardiovascular dysfunction caused by severe infection but persists after fluid resuscitation which is a subtype of sepsis with severe circulatory, cellular, and metabolic abnormalities. Sepsis and septic shock are the leading causes of morbidity and mortality among children worldwide [3]. Sepsis and septic shock are physiological and biochemical abnormalities caused by infection, which are the outcome of worsening systemic inflammatory response [4]. Sepsis and its resulting organ dysfunction are one of the leading causes of child death worldwide [5, 6]. Globally, it is estimated that the annual incidence of neonatal sepsis is 3 million cases and 1.2 million cases of children, placing a huge burden on society and families [7]. Sepsis is also an important cause of child death and disability [8]. Although there has been some improvement in the use of critical technology and monitoring and treatment, the neonatal and child mortality rate caused by sepsis is still as high as 32% in low- and middle-income countries [9]. High-income countries are still around 19%. Even in the United States, the annual incidence of sepsis is relatively high, with about 3 sepsis in every 1000 children claiming about 4500 young lives each year [10]. Most children die of sepsis suffering from refractory shock and/or multiple organ dysfunction syndrome (MODS), many of which occur within the first 48 to 72 hours of treatment [11]. Therefore, early identification, proper resuscitation, and management are very important to enhance the prognosis of children with sepsis.

The initial host immune response in children with sepsis is characterized by proinflammatory response, which can be characterized by fever, tachycardia, shortness of breath, capillary leakage, and organ dysfunction [12]. At present, C-reactive protein, procalcitonin, and interleukin-6 are the most commonly adopted biomarkers of sepsis, and their severity and prognosis are of high value in clinical research [13, 14]. However, there is also an anti-inflammatory response, which can cause changes in the process of apoptosis of various immune cells, resulting in low reactivity of innate/adaptive immune cells, which is called immune paralysis [15]. Cardiac dysfunction is a very common complication in patients with sepsis and septic shock. Studies have indicated that about 40-50% of patients with sepsis have myocardial inhibition [16]. Inflammatory factors produced by patients with sepsis, such as tumor necrosis factor-*α* and interleukin-1 *β*, mediate cardiomyocyte apoptosis and cleavage of cTnI and cTnT by regulating the activation of enzymes, resulting in the increase of troponin in the blood. Peroxides released by leukocytes during sepsis can also cause the destruction of cardiomyocytes and cause troponin elevation. In septic shock, local myocardial ischemia and hypoxia caused by microcirculatory changes will also lead to the destruction of cardiomyocytes [17]. In addition, a number of studies suggest that the increase of troponin may be related to left ventricular dysfunction, and troponin may independently predict the prognosis of patients with sepsis, but some studies also hold the opposite argument [18]. There are some differences in the methodology of these studies, such as the type of troponin, the time window for the assay, the threshold value, the experimental design, and the sample size, all of which may lead to different results [19]. It can be noticed that the increase of troponin is an important hint of cardiac dysfunction in patients with sepsis, and its value in judging the prognosis of sepsis is also worthy of further study.

Because of the nonspecific clinical manifestations of sepsis in children, its differential diagnosis is difficult. At present, the widely adopted score is Sequential Organ Failure Score (SOFA). As a means to identify septic patients, the relationship between Sequential Organ Failure Score (SOFA) and death risk has been fully verified [20]. The SOFA score needs to be tested in the laboratory; so, it cannot quickly capture the dysfunction of individual organ systems. Since the occurrence and development of sepsis is a complex pathophysiological process, a biomarker is unlikely to identify sepsis and its severity in the early stage. Future studies may include biomarkers of special significance for sepsis identification or prognosis in different categories of patients. Therefore, sepsis screening tools should include an identification kit to help clinicians' diagnosis and treatment. Based on this, this paper discusses180 children with sepsis treated in ICU from March 2019 to June 2021 in our hospital.

## 2. Patients and Methods

### 2.1. General Information

180 children with sepsis cured in ICU from March 2019 to June 2021 were enrolled as subjects and 100 children with general infection who did not meet the diagnostic criteria of systemic inflammatory response syndrome (SIRS) as controls. In the sepsis group, the age was 40 d~ 5 years (mean age of 1.03 ± 0.26 years) including 87 males and 67 females. The distribution of primary diseases included severe pneumonia (*n* = 88), intracranial infection (*n* = 54), severe hand-foot-mouth disease (*n* = 20), acute gastroenteritis with severe dehydration (*n* = 14), and others (*n* = 4). In the control group, the age was 30 d~ 4 years (mean age of 1.28 ± 0.56 years) including 59 males and 41 females. Distribution of primary diseases was as follows: 44 cases of severe pneumonia, 24 cases of intracranial infection, 12 cases of severe hand, foot, and mouth disease, 13 cases of acute gastroenteritis with severe dehydration, and 7 cases of other cases. There exhibited no significant difference in sex, age, and constituent ratio of primary disease. 29 cases died during hospitalization and follow-up, including 26 cases in sepsis group and 3 cases in the control group. The case fatality rate in the sepsis group was 14.44% (26/180) and that in the control group was 3.00% (3/100). This study was permitted by the Medical Ethics Association of our hospital, and all patients noticed informed consent.

Selection criteria were as follows: (1) patients with critical illness score ≤ 90 in PICU, (2) those who met the diagnostic criteria of 2016 International Sepsis Guidelines [21], (3) agreed to receive continuous follow-up and were able to accept and answer telephone followers, and (4) patients with complete clinical data.

Exclusion criteria were as follows: (1) patients with severe cardiac, hepatic, renal insufficiency, and malignant tumors; (2) excluding children with heart diseases after cardiac surgery, cardiopulmonary resuscitation, defibrillation, and previous heart diseases; (3) patients who refused to participate, (4) excluding children who failed to complete the relevant examination and discharge automatically after admission to PICU; (5) patients with simple virus infection; and (6) the hospitalization time ≤ 24 hours.

### 2.2. Treatment Methods

After admission, systematic physical examination, blood pressure, urine output, ECG monitoring, blood oxygen saturation, blood gas analysis, blood routine, electrolyte monitoring, and ECG examination were performed. SFOA score was performed immediately after admission to PICU, and the presence of multiple organ dysfunction syndrome (MODS) was dynamically observed. The principle of myocardial enzyme detection was as follows: after admission to PICU, 24-72 hours and before transfer to other department for treatment or transfer out of PICU and test at any time when the condition worsens.

### 2.3. Observation Indicator

#### 2.3.1. Main Outcome Indicators

The survival and death of the children 30 days after discharge were followed up through the telephone number registered at the time of admission. The outcome of the case lost by telephone was classified as illness and death.

#### 2.3.2. Myocardial Enzyme Detection

CK-MB was determined by the enzymatic method, and cTnI was determined by enzyme-labeled immunoassay. In this study, only the CK-MB and cTnI data at the first and 24-72 h after admission to PICU were enrolled as myocardial enzymatic observation indicators. Normal values were as follows: CK-MB: 0 ~ 24 U/L and cTnI 0 ~ 0.15 ng/ml, which is higher compared to the upper limit of normal values.

#### 2.3.3. Sequential Organ Failure Assessment Score **(**SOFA Scoring**)**

The SOFA score included the evaluation of respiratory, coagulation, liver, cardiovascular, neurological, and renal functions. The range of each score was 0-4. Any organ function score ≥ 2 was diagnosed as organ dysfunction, and ≥ 3 was diagnosed as organ failure.

#### 2.3.4. Other Indicators Related to Septic Death

Review the indicators related to sepsis death obtained in the literature and the medical history to collect and analyze the data of the first test after admission to PICU.

#### 2.3.5. Grouping

According to the diagnostic criteria of pediatric sepsis, patients were assigned into the sepsis and nonsepsis group. According to the survival outcome of discharge and 30 days after discharge, the patients were assigned into the death subgroup and survival subgroup, and in view of the direct correlation between SFOA score and mortality, the patients were assigned into SFOA score ≥ 2 subgroup and < 2 subgroup according to the cut-off value of SFOA score 2 set in this study.

### 2.4. Statistical Analysis

The measurement data are presented in terms of ($\bar{x}\pm s$) or median. *t*-test or *χ*^2^ test was adopted in single factor analysis of variance. The levels of CK-MB, cTnI, SOFA score, and prognosis were assessed by COX proportional hazard regression. Survival analysis was performed using Kaplan-Meier and log-rank tests, and receiver operating curve (ROC) was adopted to predict the evaluation value. *P* < 0.05 was considered statistically significant.

## 3. Results

### 3.1. Independent Risk Factors Associated with Death in Children with Sepsis

Firstly, we conducted a univariate analysis of the risk factors related to death in children with sepsis, the prognosis of children with sepsis was correlated with abnormal levels of CK-MB and cTnI, SOFA score, oxygenation index < 200, mean arterial pressure, and GCS coma score, and the difference was statistically significant (*P* < 0.05). All the results are indicated in Table 1.

### 3.2. COX Regression Analysis of Prognostic Risk Factors in Children with Sepsis

We conducted a COX regression analysis on the prognostic risk factors of children with sepsis. The results indicated that the variables with statistical significance with the death of children from sepsis were CK-MB, elevated cTnI levels, SOFA score ≥ 2, and serum. There were significant correlations between cTnI and/or CK-MB levels and SOFA score (*r* = 0.453, *P* < 0.05). All results are indicated in Table 2.

### 3.3. Comparison of Myocardial Enzyme Levels between the Sepsis and Control Groups

We compared the levels of myocardial enzymes in the sepsis and the nonsepsis group. The levels of CK-MB and (or) cTnI augmented in 121/180 cases (67.22%) in the sepsis group and in 19/198 cases in the nonsepsis group. 100 cases (19.00%) had augmented levels of CK-MB and (or) cTnI. The levels of CK-MB and cTnI in the sepsis group at the time of ICU admission and 24-72 h after admission were remarkably higher compared to the nonsepsis group. The levels of CK-MB and cTnI at 24-72 hours in the two groups were higher compared to the ICU. All the results are indicated in Table 3.

### 3.4. Comparison of Myocardial Enzyme Levels in Septic Patients with Different SFOA Scores and Survival Outcome Subgroups

We compared myocardial enzyme levels in different SFOA scores and survival outcome subgroups in the sepsis group. The subgroup with SFOA score ≥ 2 points had remarkably higher levels of CK-MB and (or) cTnI than the subgroup with SFOA score < 2 points, and the CK-MB subgroup in the survival subgroup had remarkably higher levels. The levels of -MB and (or) cTnI were remarkably higher compared to the death subgroup. The levels of CK-MB and cTnI in each subgroup at 24-72 h were remarkably higher compared to the ICU, and the difference was statistically significant (*P* < 0.05). All the results are indicated in Figures 1 and 2.

### 3.5. Survival Analysis of SFOA Score Combined with Myocardial Enzyme Level in Sepsis Group

We analyzed the survival of patients with sepsis according to SFOA score and myocardial enzyme level and assigned the levels of CK-MB and/or cTnI into normal and abnormal SFOA score ≥ 2 and< 2, respectively: (1) SFOA score ≥ 2 and CK-MB and/or cTnI augmented (group 1), (2) APSFOA score ≥ 2 and CK-MB and/or cTnI level (group 2); (3) SFOA score < 2 and CK-MB and/or cTnI augmented (group 3), and (4) SFOA score < 2 and CK-MB and/or cTnI levels were normal (group 4). Kaplan-Meier method and log-rank test were adopted for survival analysis. The survival rates of groups 1 to 4 at 30 days were 33.23%, 78.71%, 40.03%, and 100.00%, respectively. The average survival time and their 95% CI were 12.82 d (10.52~ 16.26 d), 22.34 d (18.76~ 25.81 d), 14.65 d (11.62~ 16.38 d), and 30 d (30.00~ 30.00d), respectively. Pairwise comparison between groups indicated that the survival time of children in group 1 was the shortest, and that in group 4 was the longest.

### 3.6. Evaluation Value of CK-MB, cTnI, and SOFA Score in the Definition of Sepsis 3.0 in Severe Children

The results of ROC curve showed that the scores of CK-MB, cTnI, and SOFA were 0.778 (95% CI 0.642~0.914), 0.736 (95% CI 0.602~0.890), 0.848 (95% CI 0.733~0.963), and 0.934 (95% CI 0.854~0.999), respectively. The AUC of combined diagnosis was remarkably higher compared to single factor prediction, and the difference was statistically significant (*P* < 0.05). Predictive value was displayedjoint test > SOFA score > CK − MB > cTnI. The details were displayed in Figure 3.

## 4. Discussion

Sepsis is defined as systemic inflammatory response syndrome caused by infection (suspected or confirmed) [21]. According to the national conditions of our country, experts from the first Aid Group of Pediatrics Branch of Chinese Medical Association and the Pediatric Division of Emergency Medicine in 2015 integrated and revised the recommended scheme for the diagnosis and treatment of pediatric sepsis and septic shock in China and put forward an updated version of the consensus of Chinese experts.

The most obvious infection site of sepsis is the respiratory tract, and the most common type of organ failure in sepsis is respiratory failure [22]. The etiology of sepsis varies according to geographical location, and the etiology of sepsis is complex. Pathogens may include single bacterial, viral, mycoplasma, fungal infection, or mixed infection. The clinical manifestations are diverse, and the specificity is not obvious [23]. The typical symptoms of sepsis are systemic inflammatory responses to infection, such as fever, tachycardia, shortness of breath, capillary leakage, and organ dysfunction [24]. However, there is also an anti-inflammatory response, which can cause changes in the process of apoptosis of a variety of immune cells, resulting in low reactivity of innate/adaptive immune cells. More literatures have shown that the compensatory state of immunosuppression is often accompanied by sepsis [25]. Immunosuppression caused by sepsis can affect the innate and adaptive immunity of the immune system, which may represent a combination of endogenous (such as cytokines) and exogenous (such as drugs) effects. Some epidemiological investigations show that the case fatality rate of sepsis is 25% and 80% [26]. American epidemiological data has suggested that the fatality rate of children with sepsis is 22.8%. The fatality rate of children with tumor complicated with sepsis is even as high as 68%. In recent years, SOFA score has been widely adopted as the mean to identify patients with sepsis, and the relationship between SOFA and death risk has been fully verified [27]. SOFA score indicators (such as creatinine or bilirubin levels) need to be tested in the laboratory; so, they cannot quickly capture the dysfunction of individual organ systems. The pathophysiology of sepsis is so complex that a biomarker is unlikely to identify sepsis early and assess its severity. Therefore, there is an urgent need for a simple method to identify sepsis and septic shock by combining a variety of biomarkers in clinical work.

CTnI is a highly sensitive and specific myocardial injury marker, which can be detected in serum within hours of onset [28]. The systemic inflammatory response in early sepsis is serious, which can cause cell damage and sequential and progressive organ dysfunction, induce multiple organ failure, increase oxygen consumption of stress tissue cells, and damage cardiomyocytes. Under endotoxin stimulation, tissue cells release a large number of inflammatory factors and mediators for affecting cardiomyocyte energy metabolism, directly damaging cardiomyocytes and increasing cTnI levels [29]. Some studies have indicated that the increase of cTnI level indicates that patients with sepsis have cardiac dysfunction and poor prognosis. David suggested the elevated levels of CK-MB and cTnI in patients with septic shock [30]. In recent years, it has been found that the increase of myocardial enzyme level not only reflects the injury of ischemic myocardial disease but also indicated myocardial injury and poor prognosis of noncardiogenic diseases such as sepsis [31]. Abnormal myocardial enzymes may suggest that myocardial injury “without early intervention” can rapidly develop into cardiac dysfunction and heart failure, thus inducing MODS. The results of this study indicated that the level of CK-MB or cTnI in the sepsis death subgroup was higher compared to the survival subgroup at admission to ICU and 24-72 hours after admission, suggesting that it may be an effective index to evaluate the prognosis. The increase of serum cTnI level is related to the following points: (1) mitochondrial dysfunction and organ dysfunction caused by sepsis. Mitochondrial dysfunction can mediate cardiomyocyte apoptosis and promote abnormal myocardial energy metabolism. Persistent hypoxia-ischemia caused by microcirculatory dysfunction will decrease the activity of mitochondrial electron transport complex and cytochrome C oxidase and produce a large number of reactive oxygen species [32]. Reactive oxygen species can damage the integrity of mitochondrial cell membrane, promote the disorder of intracellular calcium regulatory system, and damage the ultrastructure of myocardial mitochondria. (2) Endotoxin mediators and inflammatory mediators are released. Interleukin (IL)-6, IL-1, and tumor necrosis factor- (TNF-) *α* are the main myocardial inhibitory factors, which can promote the activation of myocardial contractile protein hydrolase and degrade myocardial contractile protein. (3) Sepsis releases a large amount of catecholamine, stimulates cardiomyocyte *β*-receptor, and increases heart rate, and persistent tachycardia will cause cardiomyocyte calcium overload and myocardial necrosis, a large amount of cTnI is released into the blood, and the level of cTnI will increase with the severity of sepsis. In this study, the factors related to the prognosis of the disease were objectively reflected by the establishment of COX model and multiple regression analysis to eliminate the confusion among the research factors. The results indicated that the factors related to the death of children with sepsis were the augmented levels of CK-MB and cTnI and the score of SOFA ≥ 2.

In the process of sepsis, the effective perfusion of various organs lessened, and the tissue cells were damaged by ischemia and hypoxia [33]. The poor tolerance of the heart to ischemia and hypoxia has become the main target organ of sepsis complicated with MODS and myocardial injury in children with sepsis can be up to 40%. In this study, the incidence of abnormal myocardial enzymes in children with sepsis was remarkably higher compared to children with nonsepsis, and the level of myocardial enzymes in children with sepsis was also remarkably higher compared to the nonsepsis group, suggesting that there might be myocardial injury in children with sepsis.

SOFA score is a clinical means to identify the severity of sepsis, and its cardiovascular score may be affected by iatrogenic intervention [34]. However, the SOFA score has been widely adopted in adult intensive care units, and the relationship between the score and the risk of death has been fully verified. Adult studies have indicated that the higher the SOFA score, the higher the mortality. In the general hospital population suspected of infection, when SOFA score is more than 2, the in-hospital mortality rate can exceed 10%. Even if the patient showed mild dysfunction, it may further worsen [35]. David and other studies found that the SOFA score of children with sepsis with long hospitalization days was remarkably higher compared to children with short hospitalization days. In addition, the SOFA score of unhealed or dead children was remarkably higher compared to enhanced or cured groups [36]. In children, SOFA scores are also remarkably higher. The SOFA score is seen as a great significance in our study, and it is a vital basis for predicting septic shock and prognosis. We can practice the SOFA score in clinical practice and optimize the score of each organ system to formulate corresponding clinical interventions measures to enhance patient outcomes. The results of this study indicated that the SOFA score was remarkably positively correlated with the levels of CK-MB and cTnI in children with sepsis with the severity of the disease. There were significant differences in the levels of CK-MB or cTnI at different time points between the SOFA score < 2 subgroup and the ≥2 subgroup, and the difference was statistically significant (*P* < 0.05).

In this study, survival analysis was conducted by combining SOFA score with CK-MB and cTnI levels. The shortest survival time was found in children with SOFA score ≥ 2 and elevated CK-MB and/or cTnI levels. The survival time of children with SOFA score < 2 and normal CK-MB and/or cTnI was the longest, suggesting that both of them had predictive value, but the predictive value of SOFA score may be greater. SOFA score combined with myocardial enzymes is helpful to judge the prognosis of sepsis. Furthermore, ROC curve was adopted to analyze the value of CK-MB, cTnI, and SOFA score in the evaluation of sepsis in critically ill children. The results indicated that the scores of CK-MB, cTnI, SOFA, and the AUC of combined detection were 0.778 (95% CI 0.642~ 0.914), 0.736 (95% CI 0.602~ 0.890), 0.848 (95% CI 0.733~ 0.963), and 0.934(95% CI 0.854~ 0.999), respectively. The AUC of combined diagnosis was remarkably higher compared to single factor prediction, and the difference was statistically significant (*P* < 0.05). Predictive value was as follows: joint test > SOFA score > CK − MB > cTnI. There are some limitations in this study. First, the sample size of this study is not large, and it is a single-center study; so, bias is inevitable. In future research, we will carry out multicenter, large-sample prospective studies, or more valuable conclusions can be drawn.

In conclusion, the increase of serum cTnI and CK-MB levels is related to the prognosis of children with sepsis, which combined with SOFA score that is helpful to judge the prognosis of sepsis.

## Figures and Tables

**Figure 1:** Comparison of CK-MB and cTnI levels at different time points between SFOA score ≥ 2 subgroup and SFOA score < 2 subgroup.

**Figure 2:** Comparison of CK-MB and cTnI levels at different time points between the survival subgroup and death subgroup.

**Figure 3:** Evaluation of ROC curve of sepsis in critically ill children by CK-MB, cTnI, and SOFA scores.

**Table 1:** Univariate analysis of mortality in patients with sepsis.

Grouping	Survival group (*n* = 154)	Death group (*n* = 26)	*t/χ* ^2^	*P*
Age (years)	4.53 ± 3.45	3.98 ± 2.51	1.294	>0.05
Gender (male/female)	95/59	18/8	0.542	>0.05
Temperature (°C)	38.45 ± 1.08	38.83 ± 2.45	1.796	>0.05
SOFA score (points)	3.16 ± 1.03	8.75 ± 2.14	29.342	<0.05
CRP (mg/L)	110.82 ± 51.27	117.93 ± 63.45	0.976	>0.05
WBC (10^9^/L)	15.26 ± 5.71	16.68 ± 7.94	1.668	>0.05
HCT (%)	31.66 ± 6.98	33.19 ± 6.58	1.682	>0.05
Na^+^ (mmol/L)	132.72 ± 8.44	133.36 ± 8.65	0.568	>0.05
K^+^ (mmol/L)	4.06 ± 0.93	4.15 ± 0.83	0.753	>0.05
Oxygenation index < 200 (*n*/%)	77 (50.00)	19 (73.07)	4.760	<0.05
Mean pulsating pressure (mmHg)	67.83 ± 15.38	42.64 ± 10.22	13.488	<0.05
Mechanical ventilation time (h)	65.52 ± 20.53	70.67 ± 45.51	1.300	>0.05
Action time of vasoactive drugs (h)	60.95 ± 30.28	68.16 ± 45.27	1.545	>0.05
GCS score (points)	12.66 ± 1.52	8.19 ± 1.36	22.860	<0.05
CM-MB and cTnI abnormalities (*n*/%)	34 (22.07)	23 (88.46)	45.301	<0.05

**Table 2:** COX regression analysis of prognostic risk factors in children with sepsis.

Variable	*B*	SE	Exp (*B*)	*P*
Oxygenation index < 200	-0.016	0.008	1.226	>0.05
SOFA score ≥ 2 points	0.778	0.312	2.083	<0.05
Mean pulsating pressure < 60 mmHg	-0.026	0.013	1.487	>0.05
GSC score < 9 points	-0.015	0.005	1.024	>0.05
CM-MB and cTnI abnormalities	0.862	0.336	2.262	<0.05

**Table 3:** Comparison of CK-MB and cTnI levels at different time points after admission between the sepsis and nonsepsis groups ($\bar{x}\pm s$).

Grouping			Sepsis group (*n* = 180)	Nonsepsis group (*n* = 100)	*P*
CK-MB normal group (*n* = 238)	CK-MB	When joining the group	13.24 ± 4.31	9.42 ± 3.56	<0.05
		24~ 72 h after admission	20.13 ± 10.11	15.45 ± 8.73	<0.05
	cTnI	When joining the group	0.06 ± 0.03	0.04 ± 0.01	<0.05
		24~ 72 h after admission	0.13 ± 0.05	0.08 ± 0.04	<0.05
CK-MB abnormal group (*n* = 140)	CK-MB	When joining the group	32.41 ± 12.78	21.54 ± 10.82	<0.05
		24~ 72 h after admission	50.67 ± 25.51	34.26 ± 14.33	<0.05
	cTnI	When joining the group	0.87 ± 0.21	0.15 ± 0.09	<0.05
		24~ 72 h after admission	1.53 ± 0.51	0.88 ± 0.33	<0.05

## Data Availability

The datasets used and analyzed during the current study are available from the corresponding author upon reasonable request.
